# Comparative Evaluation of the Treatment of COVID-19 with Multicriteria Decision-Making Techniques

**DOI:** 10.1155/2021/8864522

**Published:** 2021-01-22

**Authors:** Figen Sarigul Yildirim, Murat Sayan, Tamer Sanlidag, Berna Uzun, Dilber Uzun Ozsahin, Ilker Ozsahin

**Affiliations:** ^1^Health Science University, Antalya Education and Research Hospital, Department of Infectious Diseases and Clinical Microbiology, Antalya 07050, Turkey; ^2^Faculty of Medicine, Clinical Laboratory, PCR Unit, Kocaeli University, Kocaeli, Turkey; ^3^DESAM Institute, Near East University, 99138 Nicosia/TRNC, Mersin 10, Turkey; ^4^Department of Medical Microbiology, Manisa Celal Bayar University, Manisa, Turkey; ^5^Department of Mathematics, Near East University, 99138 Nicosia/TRNC, Mersin 10, Turkey; ^6^Department of Biomedical Engineering, Faculty of Engineering, Near East University, 99138 Nicosia/TRNC, Mersin 10, Turkey

## Abstract

**Objectives:**

The outbreak of coronavirus disease 2019 (COVID-19) was first reported in December 2019. Until now, many drugs and methods have been used in the treatment of the disease. However, no effective treatment option has been found and only case-based successes have been achieved so far. This study aims to evaluate COVID-19 treatment options using multicriteria decision-making (MCDM) techniques.

**Methods:**

In this study, we evaluated the available COVID-19 treatment options by MCDM techniques, namely, fuzzy PROMETHEE and VIKOR. These techniques are based on the evaluation and comparison of complex and multiple criteria to evaluate the most appropriate alternative. We evaluated current treatment options including favipiravir (FPV), lopinavir/ritonavir, hydroxychloroquine, interleukin-1 blocker, intravenous immunoglobulin (IVIG), and plasma exchange. The criteria used for the analysis include side effects, method of administration of the drug, cost, turnover of plasma, level of fever, age, pregnancy, and kidney function.

**Results:**

The results showed that plasma exchange was the most preferred alternative, followed by FPV and IVIG, while hydroxychloroquine was the least favorable one. New alternatives could be considered once they are available, and weights could be assigned based on the opinions of the decision-makers (physicians/clinicians). The treatment methods that we evaluated with MCDM methods will be beneficial for both healthcare users and to rapidly end the global pandemic. The proposed method is applicable for analyzing the alternatives to the selection problem with quantitative and qualitative data. In addition, it allows the decision-maker to define the problem simply under uncertainty.

**Conclusions:**

Fuzzy PROMETHEE and VIKOR techniques are applied in aiding decision-makers in choosing the right treatment technique for the management of COVID-19.

## 1. Introduction

Since December 2019, when coronavirus disease (COVID-19) incidents were first reported in Wuhan, China, an increasing number of cases have been reported in all countries on all continents except Antarctica. It exceeded the rate of the number of COVID-19 patients, thus prompting the World Health Organization to declare COVID-19 as an epidemic [1]. The virus that causes COVID-19 is called the severe acute respiratory syndrome coronavirus 2 (SARS-CoV-2). As of December 15, 2020, there were around 71,000,000 confirmed cases and 1,600,000 confirmed deaths all over the world [1].

The virus is released from respiratory secretions when an infected person speaks, sneezes, or coughs. When other people come into direct contact with these droplets, they become infected. If those who touch the surface of the virus then touch the mouth, nose, and eyes, the infection can be transmitted to other people [2–4]. The exact incubation time is unknown. It is assumed that it is between 2 and 14 days after exposure, and most cases occur within 5 days after exposure [5, 6]. Often most infections are self-limited. It may cause more serious illness in the elderly population and those with underlying medical disease [7]. According to current statistics, the most common clinical features at the onset of illness are fever in 88%, fatigue in 38%, dry cough in 67%, myalgias in 14.9%, and dyspnea in 18.7% [8]. Pneumonia is the most common complication. Severe cases have a mortality rate of 2.3 to 5% [7].

To date, there are no proven specific treatments for patients with the new virus other than supportive care. In China, Italy, France, Spain, Turkey, and now the USA, a large number of patients have received off-label and compassionate use therapies [1]. Therefore, various options have been used to fight the virus so far. Three general methods are used, including current broad-spectrum drugs, immunoenhancement therapy, and viral-specific plasma globulin. Many drugs such as chloroquine, hydroxychloroquine, azithromycin, interferon (IFN), favipiravir (FPV), remdesivir, and lopinavir/ritonavir have been used in patients with SARS or Middle East respiratory syndrome (MERS), but the effectiveness of some drugs remains controversial [9–15]. Synthetic recombinant interferon *α*, intravenous immunoglobulin (IVIG) (an immunomodulator), tocilizumab, and interleukin-1 blocker are used in immunoenhancement therapy [13, 14, 16]. Convalescent plasma therapy was thought to be an effective way to alleviate the course of the disease for seriously infected patients, and successful results were obtained in patients on whom this treatment was attempted [17, 18].

These treatment methods have largely been administered in an uncontrolled manner, with the exception of a few randomized trials launched in China and recently in the USA [19]. Hence, it is not possible to make the interpretation that if the patient dies, they die from the disease, but if the patient survives, this is because of the drug given. All methods have some advantages and disadvantages. For example, chloroquine/hydroxychloroquine, azithromycin, and lopinavir-ritonavir have several negative effects, including QT prolongation, hepatitis, acute pancreatitis, neutropenia, and anaphylaxis [20, 21]. Agents that have been used less frequently in the past (e.g., remdesivir) can cause serious negative effects that have not been detected previously due to the limited number of exposed patients [22, 23]. Interleukin blockers may cause immunosuppression, increasing the risk of sepsis, bacterial pneumonia, and hepatotoxicity [24, 25].

The rapid and simultaneous combination of supportive care and randomized control studies is the only way to find effective and safe treatments for COVID-19 and other future outbreaks. In one open-label nonrandomized control study, FPV had significantly better outcomes for disease progression and viral clearance; these results should provide an important advance in creating standard treatment guidelines for combating SARS-CoV-2 infection [26].

Decision-making models are the supportive systems that will give the necessary information to decision-makers about the alternatives and their features. PROMETHEE and VIKOR techniques are commonly used analytical multicriteria decision-making techniques that rank the alternatives under the conflicting criteria successfully applied in many fields among the other techniques. VIKOR method ranks alternatives giving the compromise solution, which is the closest to the ideal solution. PROMETHEE method gives a comparison to the alternatives based on the pairwise comparison. As opposed to other methods, PROMETHEE gives more choices to the decision-maker for defining the preference function for each criterion specifically. This makes the PROMETHEE method more sensitive in ranking the alternatives.

After the fuzzy set theory has been proposed and defined by Zadeh in 1965, the hybrid models of the classical models, fuzzy-based models, have been studied by researchers in many fields. Since there is no crisp difference between many objects and cases in the real world, it has been obtained that defining and modeling the problems using fuzzy sets can create a more sensitive model to real-world problems. And fuzzy-based MCDM techniques allow the decision-makers to analyze the alternatives even with linguistic data; it is more suitable for many cases where the numerical data are not available.

Fuzzy logic has shed light to integrate human opinion into decision-making problems [27]. In 2000, Warren et al. [28] showed the applicability of the fuzzy logic in modeling the vagueness of the treatment based on the clinical guideline knowledge to support the decision-makers in clinical practices. In 2012, Consenza [29] proposed the fuzzy expert system to provide the optimal amount of the insulin unit that should be taken before the meal for the type-1 diabetes patients corresponding to the characteristic of the food. In 2017, Santini et al. [30] proposed a fuzzy-based tool in order to manage and monitor the clinical status of *β*-thalassemia patients. This study has given exemplary results on the online determination of iron overload while monitoring the health conditions of *β*-thalassemia patients. In 2019, Akram and Adeel [31] discussed the hybrid model of the hesitant m-polar fuzzy sets. They provided the application of the hesitant m-polar fuzzy TOPSIS technique to rank and select the best alternative under m-polar fuzzy set positive and negative ideal solution for a multicriteria group decision. In 2020, Akram et al. [32] proposed Dombi aggregation operators for decision-making under m-polar fuzzy information. They tested their operation validity for obtaining the best agricultural land and the best bank with its performance. They also compared their technique with the ELECTRE-I method and they found that the optimal alternative is the same by applying the ELECTRE-I method. Garg et al. [27] proposed a new fuzzy operation compared with the Yager operation for Fermatean fuzzy numbers, and they applied this technique to obtain a ranking result for the COVID-19 testing facilities. In 2020, Akram et al. [33] presented new aggregation operators such as Fermatean fuzzy Einstein weighted averaging, Fermatean fuzzy Einstein ordered weighted averaging, generalized Fermatean fuzzy Einstein weighted averaging, and generalized Fermatean fuzzy Einstein ordered weighted averaging to cumulate the Fermatean fuzzy data in decision-making environments which has more flexible structure than the intuitionistic and Pythagorean fuzzy sets. They applied these techniques for the COVID-19 sanitizer selection problem.

Thus far, we have used a multicriteria decision-making (MCDM) technique called fuzzy PROMETHEE to compare the confusion regarding the choice of effective treatment practices using the following guidelines, to make a mutual comparison between selected treatment methods, and to determine the strongest one [34–38]. The PROMETHEE technique was developed by Brans and Vincle in 1985 [39]. Since then, it has been used successfully as an MCDM technique in many fields [40], and recently, it has been applied in the field of material selection, medicine, and healthcare [41–50], as well as it was selected as a proper COVID-19 diagnosis tool [51]. VIKOR is another commonly used MCDM technique that determines the order of alternatives under conflicting criteria based on the closeness to the ideal solution [52]. It provides the maximum group utility and the minimum individual regret for determining the compromise solution of the decision-making problem. Fuzzy logic was first presented in 1965 by Zadeh in order to define vague conditions or linguistic data mathematically [53]. A fuzzy logic-based clinical decision support system for the evaluation of renal function in posttransplant patients has been implemented successfully [54]. The analytic hierarchy process (AHP), which is another methodology based on both mathematical and psychological approaches with a similar purpose as PROMETHEE and VIKOR, is exploited to analyze and solve complex problems, in order to make the best decision. Some examples of the application of AHP in healthcare and health technologies can be found in [55–57].

The data of the COVID-19 treatment techniques contain quantitative and qualitative data of multicriteria with different importance weights which cannot be simply evaluated by the decision-makers. Therefore, we have applied two of the successfully used analytical MCDM techniques. Both of the techniques give consistent ranking results as expected. Besides, by applying the PROMETHEE method, we are able to see the positive and negative sides of each alternative.

In this study, the use of fuzzy scale based on fuzzy logic has enabled the experts to express qualitative data such as side effects, applicability, and compliance of COVID-19 treatment techniques meaningfully to be included in the model. It is also used to express the degrees of importance assigned to the criteria more easily and with the common sense of the experts.

## 2. Methods

SARS-CoV-2 is an enveloped, positive, single-strand RNA beta-coronavirus and is structurally similar to SARS-CoV-1 and MERS [58]. There are two overlapping hypotheses in the pathogenesis of the disease: triggered by the virus itself and the host response. There is significant confusion regarding the therapeutic approaches used in COVID-19. Currently, it is imperative to distinguish between the phase of viral pathogenicity and the phase in which the host inflammatory response is predominant in terms of the timing of the agent to be used in the treatment. In this case, different methods have been used to treat COVID-19 at different stages of the disease. However, scientists and real-life data have demonstrated that it is more beneficial to start many treatments early [12].

### 2.1. Treatment Techniques

We have chosen the methods that have been most frequently used since the beginning of the COVID-19 pandemic. Chloroquine, an antimalaria drug, is the first agent used against the COVID-19 disease. It both has an immune-modulating activity and can inhibit this virus with an in vitro effect [10]. It has been proven in a clinically controlled study that chloroquine, an antimalarial drug, is effective in the treatment of patients with COVID-19 [59]. Since the side effects of hydroxychloroquine are lower than chloroquine, the use of hydroxychloroquine has been preferred in the treatment of COVID-19 [60]. In COVID-19 patients, hydroxychloroquine allows the viral nasopharyngeal carriage of SARS-CoV-2 to be cleared in just three to six days [61]. Its effect is reinforced by azithromycin, an antibacterial agent [61]. Azithromycin is used to treat or prevent certain bacterial infections, predominantly those causing middle ear infections, throat, pneumonia, typhoid, bronchitis, and sinusitis [62]. Azithromycin and hydroxychloroquine have the side effect of QT prolongation (that can cause sudden death).

Remdesivir, a terminate of viral RNA transcription, has in vitro activity against SARS-CoV-2 [63]. It was originally used for the treatment of the Ebola virus disease and Marburg virus infections. One of the side effects of remdesivir is hepatotoxicity.

FPV selectively inhibits RNA-bound RNA polymerase of RNA viruses and has been approved for new influenza therapy since 2014 [64]. It is also hepatotoxic.

Lopinavir and ritonavir are antiretroviral protease inhibitors that have been used in combination for the treatment of human immunodeficiency virus infection since 2000 [65]. This has reduced the replication by 50% in the MERS coronavirus in vitro [66]. The most common side effects are gastrointestinal problems such as nausea, vomiting, and diarrhea.

Oseltamivir is a neuraminidase enzyme inhibitor used for influenza. In fact, many patients with COVID-19 symptoms might have influenza. Therefore, it is better to give this medicine to prevent the patient from getting worse [66].

Interferon is a broad-spectrum antiviral agent that acts by interacting with toll-like receptors and inhibits viral replication [67] and anti-SARS-CoV-1 activity in vitro [68].

Tocilizumab is a recombinant humanized monoclonal antibody that acts as an IL-6 receptor antagonist and is used for the treatment of rheumatoid arthritis. Interleukin-6 was reported to be released considerably in SARS and MERS patients and might play a role in the pathogenesis of these diseases [69]. In COVID-19 patients, higher plasma levels of cytokines have also been found [69].

IVIG might be the safest immunomodulator for long-term use in patients of all ages and could help to inhibit the production of proinflammatory cytokines and increase the production of anti-inflammatory mediators [13].

While evaluating these methods, we used different criteria that were selected based on the doctors, the treatment methods, and the host. Regime cost, side effects, number of tablets, dose frequency, treatment duration, plasma stability, plasma turnover, time of suppression, practicability, intravenous form, oral form, and drug-drug interaction were chosen as the treatment method-related criteria. Age, pregnancy, glomerular filtration rate (GFR), compliance, fever, pneumonia, intensive care, organ failure, macrophage activation syndrome, and the hemophagocytic syndrome were chosen as the host-related criteria. These are symptoms and phases of diseases in COVID patients. False prescription and inefficient drug combination were chosen as the doctor-related criteria. All of these factors are important when selecting treatment methods for COVID-19 patients.

### 2.2. Fuzzy-Based MCDM Models

Ranking the fuzzy numbers contains the main problematic part of the decision-making problems under the fuzzy environment. This process is also the most important stage of the decision-making process since it simplifies the complexity of the problem. Comparison of the fuzzy numbers has practical applications in optimization, forecasting, decision-making, and approximate reasoning. Real-world decision problems often involve uncertain conditions of the properties of alternatives, and fuzzy numbers allow the decision-maker to be used in the analysis by taking these uncertain conditions into account. There are many types of fuzzy-based MCDM models available for different aims, and there are many studies that present different techniques for the comparison of the fuzzy numbers [70–72]. Although the centroid concept has been applied in many fields and has been known for hundreds of years, first in 1980, Yager proposed the centroid method for the comparison of the fuzzy numbers [73]. After Yager, there have been many studies that used this method for the construction of the individually defined ranking index [74–76]. Some of these researchers have used the value of *x* alone, while some of them used a combination of *x* and *y* values to obtain their own ranking index that depends on the centroid concept. There are also some research studies that aim to produce the most suitable or correct centroid value formula [77, 78] for the usage of the ranking index. These research studies provide valuable information for comparing the fuzzy numbers that depend on the centroid approaches. However, some studies found that the Yager index has great potential in fuzzy optimization [79]. In our study, some of the criteria, such as side effects, were defined by the experts using the linguistic fuzzy scale since no crisp values are available for those criteria. Furthermore, fuzzy data of the defined parameters have been compared using the centroid concept, defined by the Yager index, which is successfully applied and confirmed by many researchers. If we could have used different fuzzy models most probably, we will obtain the same ranking results.

### 2.3. Fuzzy PROMETHEE

In real-world problems, one of the major challenges involves the collection of crisp data to analyze systems. In 1965, Zadeh laid the foundations for the idea of establishing a rule functioning and then transferring it to a machine by making use of human life experiences and various kinds of knowledge. Fuzzy logic can be defined as a decision mechanism design in its simplest form. It allows decision-makers to identify vague conditions and analyze the systems using linguistic data if it is needed [53].

MCDM is a research area that involves the analysis of various available choices in a situation or research area, which spans daily life, social sciences, engineering, medicine, and many other areas.

MCDM analyzes the alternatives (qualitatively or quantitatively) involved in a criterion that makes the alternatives a favorable or unfavorable choice for a particular application and attempts to compare this criterion based on the selected criteria against every other available option in an attempt to support the decision-maker when selecting an option with maximum advantages without negotiation.

PROMETHEE is an MCDM tool that allows a user to analyze and rank accessible alternatives according to the criteria of each alternative. It compares the available alternatives based on the selected criteria [39]. The PROMETHEE technique is a valuable and sensitive MCDM technique for reasons that include the following:

- PROMETHEE can be used to handle qualitative and quantitative criteria simultaneously
- PROMETHEE deals with fuzzy relations, vagueness, and uncertainties
- PROMETHEE is easy to handle and provides the user with maximum control over the preference of the alternatives with regard to the criteria

When using PROMETHEE, only two types of information are required from the decision-maker: information regarding the importance weights of the selected criteria and the preference function to be used in comparing the alternatives' contribution with regard to each criterion.

Different preference functions (*P*_j_) are available on PROMETHEE for the definition of different criteria. The preference function defines assigning values to the ranking of two alternatives (a and *a*_t_) in relation to specific criteria and a preference degree of the limit between 0 and 1 [39]. The preference functions for practical purposes that can be used at the discretion of the decision-maker include the usual function, V-shape function, level function, u-shape function, linear function, and Gaussian function [39]. A complete explanation of the preference functions used, their ranking, and how to make a decision on which function best suits a scenario was presented by Brans et al. [39].

In the PROMETHEE analysis, after collecting the criteria of the alternatives, the preference function *p*_j_ (d) for each criterion *j* should be defined, and the importance weight of each criterion *w*_*t*_ = (*w*_1_, *w*_2_,…, *w*_*k*_) should be determined. Normalization of the weights or equality of weights can be chosen by the decision-maker based on the application. Then, for every alternative pair (*a*_t_, *a*_t'_ ∈ A), the outranking relation *π*(*a*_*t*_, *a*_*t*′_) should be determined as seen in

(1) $$\begin{array}{c} \;\pi \left(a_{t},a_{t^{\prime }}\right)=\sum_{k=1}^{K}w_{k}.\left[p_{k}\left(f_{k}\left(a_{t}\right)-f_{k}\left(a_{t^{\prime }}\right)\right)\right],\;AXA⟶\left[0,1\right]. \end{array}$$

And the positive outranking flow of *a*_*t*_(Φ^+^(*a*_*t*_)) and the negative outranking flow of *a*_*t*_(Φ^−^(*a*_*t*_)) should be calculated as seen in

(2) $$\begin{array}{c} \Phi^{+}\left(a_{t}\right)=\frac{1}{n-1}\sum_{\begin{array}{c} t^{\prime }=1\\ t^{\prime }\neq t \end{array}}^{n}\pi \left(a_{t},a_{t^{\prime }}\right),\\ \Phi^{-}\left(a_{t}\right)=\frac{1}{n-1}\sum_{\begin{array}{c} t^{\prime }=1\\ t^{\prime }\neq t \end{array}}^{n}\pi \left(a_{t},a_{t^{\prime }}\right), \end{array}$$

where *n* denotes the number of options, and each option is compared to the *n* − 1 number of alternatives. The positive outranking flow is an illustration of how a particular alternative is greater than the other options. The higher the positive outranking flow of a particular alternative is, the greater the possibilities are. The negative outranking flow is an expression of how a particular alternative is less preferred compared to the other alternatives. The lower the negative outranking value is, the greater the alternatives are [1–9, 16]. PROMETHEE gives a partial preorder of the alternatives as seen in equation (3).

*a*_*t*_ is preferred to alternative *a*_*t*′_ (*a*_*t*_*Pa*_*t*′_) if

(3) $$\begin{array}{c} \left\{\begin{array}{c} \Phi^{+}\left(a_{t}\right)\geq \Phi^{+}\left(a_{t^{\prime }}\right)\text{ and }\Phi^{-}\left(a_{t}\right)<\Phi^{-}\left(a_{t^{\prime }}\right),\\ \Phi^{+}\left(a_{t}\right)>\Phi^{+}\left(a_{t^{\prime }}\right)\text{ and }\Phi^{-}\left(a_{t}\right)=\Phi^{-}\left(a_{t^{\prime }}\right). \end{array}\right. \end{array}$$

*a*_*t*_ is indifferent to alternative *a*_*t*′_ (*a*_*t*_*Ia*_*t*′_) if

(4) $$\begin{array}{c} \Phi^{+}\left(a_{t}\right)=\Phi^{+}\left(a_{t^{\prime }}\right)\text{ and }\Phi^{-}\left(a_{t}\right)=\Phi^{-}\left(a_{t^{\prime }}\right). \end{array}$$

*a*_*t*_ is incomparable to *a*_*t*′_(*a*_*t*_*Ra*_*t*′_) if

(5) $$\begin{array}{c} \left\{\begin{array}{c} \Phi^{+}\left(a_{t}\right)>\Phi^{+}\left(a_{t^{\prime }}\right)\text{ and }\Phi^{-}\left(a_{t}\right)>\Phi^{-}\left(a_{t^{\prime }}\right),\\ \Phi^{+}\left(a_{t}\right)<\Phi^{+}\left(a_{t^{\prime }}\right)\text{ and }\Phi^{-}\left(a_{t}\right)<\Phi^{-}\left(a_{t^{\prime }}\right). \end{array}\right. \end{array}$$

Using PROMETHEE II, the net flow of an alternative *a*_*t*_(Φ^net^(*a*_*t*_)) can be calculated with

(6) $$\begin{array}{c} \Phi^{\text{net}}\left(a_{t}\right)=\Phi^{+}\left(a_{t}\right)-\Phi^{-}\left(a_{t}\right). \end{array}$$

And the net ranking results of the alternatives can be found by

(7) $$\begin{array}{c} \left(a_{t}Pa_{t^{\prime }}\right)\text{ if }\Phi^{\text{net}}\left(a_{t}\right)>\Phi^{\text{net}}\left(a_{t^{\prime }}\right), \end{array}$$

(8) $$\begin{array}{c} \left(a_{t}Ia_{t^{\prime }}\right)\text{ if }\Phi^{\text{net}}\left(a_{t}\right)=\Phi^{\text{net}}\left(a_{t^{\prime }}\right). \end{array}$$

The better alternative is the one with the higher Φ^net^(*a*_*t*_) value (32).

In this study, we proposed the use of the fuzzy-based PROMETHEE technique for the evaluation of the available treatment options for COVID-19. The selected treatment options are favipiravir (FPV), remdesivir, “lopinavir/ritonavir,” “hydroxychloroquine,” “oseltamivir + hydroxychloroquine,” “hydroxychloroquine + azithromycin,” interleukin-1 blocker, tocilizumab, “interferon,” intravenous immunoglobulin (IVIG), and plasma exchange. The selected criteria of the alternatives and the importance weight with fuzzy scale can be seen in Table 1. The data and the weights of the criteria have been collected by the experts.

The Yager index was used for the defuzzification of the fuzzy scale. Lastly, the PROMETHEE-Gaia decision lab program with Gaussian preference functions has been used for the evaluation.

### 2.4. Fuzzy VIKOR

The basis of the VIKOR (Multicriteria Optimization and Compromise Solution) method is based on the determination of a compromise solution in the light of alternatives and within the scope of the evaluation criteria. This compromise solution has been determined as the closest solution to the ideal solution [80, 81]. With the expression of a compromise solution, it is understood that by creating a multicriteria ranking index for alternatives, the closest decision is made to the ideal solution under certain conditions. Under the assumption that each alternative is evaluated on the basis of decision-making criteria, consensus ranking is achieved by comparing the values of proximity to the ideal alternative [82]. This technique is also based on obtaining the ranking results of alternatives with maximum group benefit and therefore minimum regret of individuals.

After constructing the decision matrix of the MCM problem with specifying the importance weights of each criterion, the steps of the VIKOR method can be summarized as follows.

**Step 1 .**

(determination of the best ((*f*_*i*_*∗*) and the worst ((*f*_*i*_^−^) values of each criterion). The best values should be determined as the maximum point of beneficial criteria and the minimum point of the criteria that cause cost. If the criterion-*i* is the beneficial criterion, then *f*_*i*_*∗* and *f*_*i*_^−^ can be obtained by using the following formulas:

(9) $$\begin{array}{c} f_{i}^{*}=\underset{j}{\max}\left(f_{ij}\right), \end{array}$$

(10) $$\begin{array}{c} f_{i}^{-}=\underset{j}{\min}\left(f_{ij}\right). \end{array}$$

*f*_*ij*_ denotes the value of the *j*-th criterion of the *i*-th alternative.

**Step 2 .**

(obtaining the Utility (*S*_*i*_) and Regret (*R*_*i*_) values for each alternative). The utility (*S*_*i*_) and regret (*R*_*i*_) values of the alternative-*i* can be calculated by using the following formulas:

(11) $$\begin{array}{c} S_{i}=\sum_{i=1}^{n}w_{i}\left[\frac{f_{i}^{*}-f\left(ij\right)}{f_{i}^{*}-f_{i}^{-}}\right], \end{array}$$

(12) $$\begin{array}{c} R_{i}=\underset{j}{\max}\left(w_{i}\left[\frac{f_{i}^{*}-f\left(ij\right)}{f_{i}^{*}-f_{i}^{-}}\right]\right), \end{array}$$

where *w*_*i*_ denotes the importance weights of the criterion-*j*, which represents the relative importance degrees.

**Step 3 .**

(computing the value of *Q*_*j*_ and ranking the alternatives accordingly). *Q*_*j*_ values can be obtained based on the relation given as

(13) $$\begin{array}{c} Q_{j}=v\left[\frac{S_{j}-\text{min}\left(S_{j}\right)}{\text{max}\left(S_{j}\right)-\text{min}\left(S_{j}\right)}\right]+\left(1-v\right)\left[\frac{R_{j}-\text{min}\left(R_{j}\right)}{\text{max}\left(R_{j}\right)-\text{min}\left(R_{j}\right)}\right], \end{array}$$

where *v* ∈ [0,1] and represents the weight/level of the strategy that indicates the maximum group utility and (1 − *v*) represents the weight/level of the individual regret. The value of *v* is most commonly used as 0.5, so as in this study.

When *v* value (>0.5) is chosen high, it is stated that the majority tend to show a positive attitude toward *Q*_*j*_ index. When the *v* value (<0.5) is chosen less, it means that the majority shows a negative attitude. In general, it is assumed that the evaluation expert groups (positive and negative) have a conciliatory attitude by selecting the *y* value = 0.5 [83].

The alternative with the smallest *Q*_*j*_ value is indicated as the best option within the group of alternatives. And, the ranking can be obtained accordingly.

However, in order to consider the alternative with a minimum value of *Q*_*j*_ as the best alternative with an acceptable advantage, it must meet the following conditions:

   Condition 1 (acceptable advantage): the acceptable advantage is the existence of a significant difference between the best and the closest options, which should be calculated as
  (14) $$\begin{array}{c} Q\left(A^{\prime \prime }\right)-Q\left(A{}^{\prime }\right)\geq DQ\;. \end{array}$$
*A*′ denotes the best alternative with the minimum *Q* value and *A*^'′^ denotes the second-best alternative with the second minimum *Q*_*j*_.
  (15) $$\begin{array}{c} DQ=\frac{1}{\left(m-1\right)}, \end{array}$$
where *m* indicates the number of the alternatives.
Condition 2 (acceptable stability): *A*′ should have the minimum (best) value/s of the *R*_*j*_ and/or *S*_*j*_ between all of the alternatives.
In VIKOR, if the best alternative with the min (*Q*_*j*_) does not satisfy one of the given conditions, then the compromise solutions set can be proposed as follows:
  (i) If only condition 2 is not satisfied, one has *A*′ and *A*^'′^
  (ii) If the first condition is not satisfied, one has *A*′,  *A*^'′^, ...,  *A*^*M* ^where *M* represents the maximum decision points that meet the condition

(16) $$\begin{array}{c} Q\left(A^{M}\right)-Q\left(A^{\prime }\right)<DQ\;. \end{array}$$

## 3. Results

Table 2 shows the complete ranking results of the COVID-19 treatment options with the positive, negative, and net flow ranking of the alternatives. According to the table, plasma exchange and FVP outrank the other treatment options with net flows of 0.0268 and 0.0265, respectively, followed by IVIG. The least ranked COVID-treatment option is hydroxychloroquine with a net flow of −0.0502. Similarly, Figure 1 shows the strong and weak points of the COVID-19 treatment options.

These results of the VIKOR technique validate the ranking results of the PROMETHEE technique. Using the VIKOR method, we obtained almost the same net ranking for the selected COVID-19 treatment alternatives as seen in Table 3.

## 4. Discussion

In our study, we compared the treatment applications used in COVID-19 treatment between December 2019 and March 2020 with MCDM methods. Clinical studies of the treatment methods used are still ongoing. In our study, the plasma exchange method was found to be the best method among the treatment options, similar to clinical applications. It has been suggested that plasma from cured patients should be used for treatment [84]. Indeed, healing patients often have a high level of antibodies to the pathogen present in their blood. Antibodies are immunoglobulin produced by B lymphocytes to fight pathogens and other foreign bodies, to recognize and neutralize unique molecules in pathogens [85]. Based on this, patients who recovered from COVID-19 recovered and were injected plasma into serious patients after collection and processing, and within 24 hours, there was a decrease in inflammation and viral loads as well as an improvement in oxygen saturation in the blood [86].

FVP was found to be the second-best method of treatment for COVID-19 patients. The patients who were treated with FVP showed faster viral clearance, shorter fever period, and improvement in radiological findings in Wuhan [87]. The third best one was found to be IVIG which may also play a role in the control of the immune system, where there is a high level of inflammation. Improvement in the poor prognosis stage of the disease is poor, and IVIG can be quickly recognized and applied for this treatment [13].

When we compared the methods related to the criteria, the others were interleukin-1 blocker, remdesivir, interferon, tocilizumab, oseltamivir + hydroxychloroquine + azithromycin, lopinavir/ritonavir, oseltamivir + hydroxychloroquine, and hydroxychloroquine. These criteria are very important, not only for patients but also for treatment practitioners.

The spread of COVID-19 is continuing at a rapid pace. It is very important to discover effective treatment or prophylactic agents among measures such as staying at home, hand hygiene, wearing masks, and so on to stop the pandemic. Health professionals and the global scientific community are waiting for new evidence to emerge soon to manage COVID-19. Until this evidence emerges, it is necessary to continue using the treatment methods that have shown effectiveness. The treatment methods that we evaluated with MCDM methods will be beneficial for both healthcare users and to rapidly end the global pandemic.

In this study, an average patient was considered to show the method's applicability, so the patient profile such as gender or disease stage was not included in the analysis. However, this study can be extended to include all possible factors since fuzzy PROMETHEE and VIKOR are able to support a large number of inputs. Another limitation of this study is the fact that treatment selection might be different for patients in the acute phase than those in the stable phase which was not considered in this study.

The proposed method is applicable for analyzing the alternatives to the selection problem with quantitative and qualitative data. In addition, it allows the decision-maker to define the problem simply under uncertainty. One of the limitations of this technique is that there is no method for determining the weight of the criteria. Therefore, expert opinion is of great importance in establishing criteria weights for this model to give accurate results in practical applications.

## 5. Conclusion

In this study, we analyzed different treatment options for COVID-19 treatment using fuzzy PROMETHEE and VIKOR methods. Overall, there is no globally approved specific antiviral drug available for COVID-19. All drug options come from the experience of treating SARS, MERS, or other new influenza viruses. Active symptomatic support is the key to treatment. The above medicines will help, and their efficacy needs further confirmation. New alternatives and criteria could be considered once they are available in the future, and weights could be assigned based on the opinions of the decision-makers (physicians/clinicians). We showed the applicability of the MCDM techniques in informing decision-makers in terms of choosing the right treatment technique for the management of COVID-19.

## Figures and Tables

**Figure 1:** Positive and negative aspects of each COVID-19 treatment option. The higher the criterion stands in the graph in the positive side, the higher it contributes to the positive side of the technique. Similarly, the lower the criterion stands in the graph on the negative side, the higher it contributes to the negative side of the technique.

**Table 1:** Criteria of the COVID-19 treatment options and their importance weights with fuzzy linguistic scale.

Linguistic scale for evaluation	Triangular fuzzy scale	Importance ratings of criteria
Very high (VH)	(0.75, 1, 1)	Side effects, regime cost, number of tablets, dose frequency, treatment duration, plasma stability, plasma turnover, time of suppression, practicability, drug-drug interaction, compliance, fever, pneumonia, intensive care, organ failure, macrophage activation syndrome, hemophagocytic syndrome
Important (H)	(0.50, 0.75, 1)	Age, pregnancy, GFR
Medium (M)		Intravenous form, oral form, false prescription
Low (L)		Inefficient drug combination
Very low (VL)		-

**Table 2:** Complete ranking of COVID-19 treatment options with PROMETHEE.

Complete ranking	Options (*a*_*t*_)	Net flow Φ^net^(*a*_*t*_)	Positive flow Φ^+^(*a*_*t*_)	Negative flow Φ^−^(*a*_*t*_)
1	Plasma exchange	0.0268	0.0364	0.0095
2	Favipravir	0.0265	0.0361	0.0096
3	Intravenous immunoglobulin (IVIG)	0.0199	0.0318	0.0120
4	Interleukin-1 blocker	0.0189	0.0335	0.0135
5	Tocilizumab	0.0184	0.0342	0.0158
6	Remdesivir	0.0177	0.0340	0.0162
7	Interferon	0.0139	0.0283	0.0144
8	Oseltamivir + hydroxychloroquine + azithromycin	−0.0188	0.0165	0.0352
9	Lopinavir/ritonavir	−0.0348	0.0239	0.0588
10	Oseltamivir + hydroxychloroquine	−0.0384	0.0103	0.0487
11	Hydroxychloroquine	−0.0502	0.0108	0.0609

**Table 3:** Complete ranking of COVID-19 treatment options with VIKOR.

Complete ranking	Alternatives	Qj	Sj	Rj
1	Plasma exchange	0	5.1	0.92
2	Favipravir	0.013387978	5.345	0.92
3	Intravenous immunoglobulin	0.050273224	6.02	0.92
4	Interleukin-1 blocker	0.093442623	6.81	0.92
5	Remdesivir	0.113934426	7.185	0.92
6	Interferon	0.116393443	7.23	0.92
7	Tocilizumab	0.125136612	7.39	0.92
8	Oseltamivir + hydroxychloroquine + azithromycin	0.310382514	10.78	0.92
9	Lopinavir/ritonavir	0.337978142	11.285	0.92
10	Oseltamivir + hydroxychloroquine	0.449726776	13.33	0.92
11	Hydroxychloroquine	0.5	14.25	0.92

## Data Availability

All data generated or analyzed during this study are included within this published article.

## References

[1] World Health Organization (2020). Situation updates on March 26, 2020. https://covid19.who.int/.

[2] Rothe C., Schunk M., Sothmann P. (2020). Transmission of 2019-nCoV infection from an asymptomatic contact in Germany. *New England Journal of Medicine*.

[3] Kupferschmidt K. (2020). Study claiming new coronavirus can be transmitted by people without symptoms was flawed science. *The Journal of Infectious Diseases*.

[4] Bai Y., Yao L., Wei T. (2020). Presumed asymptomatic carrier transmission of COVID-19. *JAMA*.

[5] Li Q., Guan X., Wu P. (2020). Early transmission dynamics in wuhan, China, of novel coronavirus-infected pneumonia. *New England Journal of Medicine*.

[6] Chan J. F.-W., Yuan S., Kok K.-H. (2020). A familial cluster of pneumonia associated with the 2019 novel coronavirus indicating person-to-person transmission: a study of a family cluster. *The Lancet*.

[7] Yi Y., Lagniton P. N. P., Ye S., Li E., Xu R.-H. (2020). COVID-19: what has been learned and to be learned about the novel coronavirus disease. *International Journal of Biological Sciences*.

[8] Chen N., Zhou M., Dong X. (2020). Epidemiological and clinical characteristics of 99 cases of 2019 novel coronavirus pneumonia in Wuhan, China: a descriptive study. *The Lancet*.

[9] Holshue M. L., DeBolt C., Lindquist S. (2020). First case of 2019 novel coronavirus in the United States. *New England Journal of Medicine*.

[10] Wang M., Cao R., Zhang L. (2020). Remdesivir and chloroquine effectively inhibit the recently emerged novel coronavirus (2019-nCoV) in vitro. *Cell Research*.

[11] Gao J., Tian Z., Yang X. (2020). Breakthrough: chloroquine phosphate has shown apparent efficacy in treatment of COVID-19 associated pneumonia in clinical studies. *BioScience Trends*.

[12] Lu H. (2020). Drug treatment options for the 2019-new coronavirus (2019-nCoV). *BioScience Trends*.

[13] Gilardin L., Bayry J., Kaveri S. V. (2015). Intravenous immunoglobulin as clinical immune-modulating therapy. *Canadian Medical Association Journal*.

[14] Kumar V., Jung Y.-S., Liang P.-H. (2013). Anti-SARS coronavirus agents: a patent review (2008-present). *Expert Opinion on Therapeutic Patents*.

[15] Mustafa S., Balkhy H., Gabere M. N. (2018). Current treatment options and the role of peptides as potential therapeutic components for Middle East Respiratory Syndrome (MERS): a review. *Journal of Infection and Public Health*.

[16] Actemra (tocilizumab) (2019). Prescribing information. Genentech. https://www.actemrahcp.com/?_ga=2.%20137041460.509331555.1584929819-505112783.

[17] Mair-Jenkins J., Saavedra-Campos M., Baillie J. K. (2015). The effectiveness of convalescent plasma and hyperimmune immunoglobulin for the treatment of severe acute respiratory infections of viral etiology: a systematic review and exploratory meta-analysis. *Journal of Infectious Diseases*.

[18] Zhang L., Liu Y. (2020). Potential interventions for novel coronavirus in China: a systematic review. *Journal of Medical Virology*.

[19] Adaptive COVID-19 treatment trial (2020). ClinicalTrials.gov identifier: nct04280705. https://clinicaltrials.gov/ct2/show/NCT04280705?%20Term=remdesivir&cond=covid-19&draw=2&rank=5.

[20] Young B. E., Ong S. W. X., Kalimuddin S. (2020). Epidemiologic features and clinical course of patients infected with SARS-CoV-2 in Singapore novel coronavirus outbreak research team. Epidemiologic features and clinical course of patients infected with SARS-CoV-2 in Singapore. *Jama*.

[21] Wu Z., McGoogan J. M. (2020). Characteristics of and important lessons from the coronavirus disease 2019 (COVID-19) outbreak in China. *Jama*.

[22] Reina J. (2020). The antiviral hope against SARS-CoV-2. *Revista Española de Quimioterapia*.

[23] Kupferschmidt K., Cohen J. (2020). Race to find COVID-19 treatments accelerates. *Science*.

[24] Kalil A. C., Sun J. (2011). Low-dose steroids for septic shock and severe sepsis: the use of Bayesian statistics to resolve clinical trial controversies. *Intensive Care Medicine*.

[25] tocilizumab A. (2019). Prescribing information. Genentech. https://www.actemrahcp.com/?_ga=2.%20137041460.509331555.1584929819-505112783.%201584929819.

[26] Cai Q., Yang M., Liu D. *Experimental Treatment with Favipiravir for COVID-19: An Open-Label Control Study Engineering*.

[27] Garg H., Shahzadi G., Akram M. (2020). Decision-making analysis based on Fermatean fuzzy Yager aggregation operators with application in COVID-19 testing facility. *Mathematical Problems in Engineering*.

[28] Warren J., Beliakov G., van der Zwaag B. Fuzzy logic in clinical practice decision support systems.

[29] Cosenza B. (2012). Off-line control of the postprandial glycemia in type 1 diabetes patients by a fuzzy logic decision support. *Expert Systems with Applications*.

[30] Santini S. Using fuzzy logic for improving clinical daily-care of *β*-thalassemia patients.

[31] Akram M., Adeel A. (2019). Novel TOPSIS method for group decision-making based on hesitant m-polar fuzzy model. *Journal of Intelligent & Fuzzy Systems*.

[32] Akram M., Yaqoob N., Ali G., Chammam W. (2020). Extensions of Dombi aggregation operators for decision making under m-polar fuzzy information. *Journal of Mathematics*.

[33] Akram M., Shahzadi G., Ahmadini A. A. H. (2020). Decision-making framework for an effective sanitizer to reduce COVID-19 under fermatean fuzzy environment. *Journal of Mathematics*.

[34] Uzun B., Sarıgül Yıldırım F., Sayan M., Şanlıdağ T., Uzun Ozsahin D. (2019). *The Use Of Fuzzy Promethee Technique In Antiretroviral Combination Decision In Pediatric Hiv Treatments*.

[35] Sayan M., Sultanoglu N., Uzun B., Yıldırım F. S., Şanlıdağ T., Ozsahin D. U. (2019). *Determination of Post-Exposure Prophylaxis Regimen in the Prevention of Potential Pediatric HIV-1 Infection by the Multi-Criteria Decision-Making Theory*.

[36] Sultanoglu N., Uzun B., Yıldırım F. S., Sayan M., Şanlıdağ T., Ozsahin D. U. (2019). *Selection of the Most Appropriate Antiretroviral Medication in Determined Aged Groups (≥ 3 Years) of HIV-1 Infected Children*.

[37] Sayan M., Sanlidag T., Sultanoglu N., Uzun B., Yildirim F. S., Ozsahin D. U., Aliev R., Kacprzyk J., Pedrycz W., Jamshidi M., Babanli M., Sadikoglu F. (2020). Evaluating the efficacy of adult HIV post exposure prophylaxis regimens in relation to transmission risk factors by multi criteria decision method. *Advances in Intelligent Systems and Computing*.

[38] Sayan M., Uzun Ozsahin D., Sanlidag T., Sultanoglu N., Sarigul Yildirim F., Uzun B., Aliev R., Kacprzyk J., Pedrycz W., Jamshidi M., Babanli M., Sadikoglu F. (2020). Efficacy evaluation of antiretroviral drug combinations for HIV-1 treatment by using the fuzzy PROMETHEE. *Advances in Intelligent Systems and Computing*.

[39] Brans J. P., Vincke P. (1985). A preference ranking Organisation method: the PROMETHEE method for MCDM. *Management Science*.

[40] Asemi A., Baba M. S., Asemi A., Abdullah R., Idris N. Fuzzy multi criteria decision making applications: a review study.

[41] Ozsahin I., Abebe S., Mok G. (2020). A multi-criteria decision-making approach for schizophrenia treatment techniques. *Archives of Psychiatry and Psychotherapy*.

[42] Ozsahin I. (2020). Identifying a personalized anesthetic with fuzzy PROMETHEE. *Healthcare Informatics Research*.

[43] Ozsahin I., Uzun Ozsahin D., Maisaini M., Mok P. (2019). Fuzzy PROMETHEE analysis of leukemia treatment techniques. https://www.wcrj.net/article/1315.

[44] Ozsahin I., Uzun Ozsahin D., Nyakuwanikwa K., Wallace Simbanegav T. (2019). *Fuzzy PROMETHEE for Ranking Pancreatic Cancer Treatment Techniques*.

[45] Maisaini M., Uzun B., Ozsahin I., Uzun D. Evaluating lung cancer treatment techniques using fuzzy PROMETHEE approach.

[46] Uzun Ozsahin D., Ozsahin I. (2018). A fuzzy PROMETHEE approach for breast cancer treatment techniques. *Health Sciences*.

[47] Uzun D., Uzun B., Sani M., Ozsahin I. (2018). Evaluating X-ray based medical imaging devices with fuzzy preference ranking organization method for enrichment evaluations. *International Journal of Advanced Computer Science and Applications*.

[48] Ozsahin D., Isa N., Uzun B., Ozsahin I. Effective analysis of image reconstruction algorithms in nuclear medicine using fuzzy PROMETHEE.

[49] Ozsahin I., Sharif T., Ozsahin D. U., Uzun B. (2019). Evaluation of solid-state detectors in medical imaging with fuzzy PROMETHEE. *Journal of Instrumentation*.

[50] Taiwo Mubarak M., Ozsahin I., Uzun Ozsahin D. (2019). *Evaluation of Sterilization Methods for Medical Devices*.

[51] Sayan M., Sanlidag T., Berna U., Ozsahin I. (2020). Capacity evaluation of diagnostic tests for COVID-19 using multicriteria decision-making techniques. *Computational and Mathematical Methods in Medicine*.

[52] Zhang N., Wei G. (2013). Extension of VIKOR method for decision making problem based on hesitant fuzzy set. *Applied Mathematical Modelling*.

[53] Zadeh L. A. (1965). Fuzzy sets. *Information and Control*.

[54] Improta G., Mazzella V., Vecchione D., Santini S., Triassi M. (2020). Fuzzy logic-based clinical decision support system for the evaluation of renal function in post‐Transplant Patients. *Journal of Evaluation in Clinical Practice*.

[55] mprota G., Converso G., Murino T., Mosè G., Antonietta P., Maria R. (2019). Analytic hierarchy process (AHP) in dynamic configuration as a tool for health technology assessment (HTA): the case of biosensing optoelectronics in oncology. *International Journal of Information Technology & Decision Making*.

[56] Improta G., Perrone A., Russo M. A., Maria T. (2019). Health technology assessment (HTA) of optoelectronic biosensors for oncology by analytic hierarchy process (AHP) and Likert scale. *BMC Medical Research Methodology*.

[57] Improta G., Russo M. A., Triassi M., Converso G., Murino T., Santillo L. C. (2018). Use of the AHP methodology in system dynamics: modelling and simulation for health technology assessments to determine the correct prosthesis choice for hernia diseases. *Mathematical Biosciences*.

[58] Lu R., Zhao X., Li J. (2020). Genomic characterisation and epidemiology of 2019 novel coronavirus: implications for virus origins and receptor binding. *The Lancet*.

[59] Multicenter collaboration group of Department of Science and Technology of Guangdong Province (2020). Expert consensus on chloroquine phosphate for the treatment of novel coronavirus pneumonia. *Zhonghua*.

[60] Marmor M. F., Kellner U., Lai T. Y. Y., Melles R. B., Mieler W. F. (2016). Recommendations on screening for chloroquine and hydroxychloroquine retinopathy (2016 revision). *Ophthalmology*.

[61] Gautret P., Lagier J.-C., Parola P. (2020). Hydroxychloroquine and azithromycin as a treatment of COVID-19: results of an open-label non-randomized clinical trial. *International Journal of Antimicrobial Agents*.

[62] Bakheit A. H. H., Al-Hadiya B. M. H., Abd-Elgalil A. A. (2014). Azithromycin. *Profiles of Drug Substances, Excipients and Related Methodology*.

[63] Cao Y.-C., Deng Q.-X., Dai S.-X. (2020). Remdesivir for severe acute respiratory syndrome coronavirus 2 causing COVID-19: an evaluation of the evidence. *Travel Medicine and Infectious Disease*.

[64] Furuta Y., Takahashi K., Kuno-Maekawa M. (2005). Mechanism of action of T-705 against influenza virus. *Antimicrobial Agents and Chemotherapy*.

[65] Cvetkovic R. S., Goa K. L. (2003). Lopinavir/ritonavir. *Drugs*.

[66] Momattin H., Al-Ali A. Y., Al-Tawfiq J. A. (2019). A systematic review of therapeutic agents for the treatment of the Middle East respiratory syndrome coronavirus (MERS-CoV). *Travel Medicine and Infectious Disease*.

[67] Uematsu S., Akira S. (2007). Toll-like receptors and type I interferons. *Journal of Biological Chemistry*.

[68] Ströher U., DiCaro A., Li Y. (2004). Severe acute respiratory syndrome-related coronavirus is inhibited by interferon‐*α*. *The Journal of Infectious Diseases*.

[69] Huang C., Wang Y., Li X. (2020). Clinical features of patients infected with 2019 novel coronavirus in Wuhan, China. *The Lancet*.

[70] Yager R. (1981). A procedure for ordering fuzzy subsets of the unit interval. *Information Science*.

[71] Wang X., Kerre E. E. (2001). Reasonable properties for the ordering of fuzzy quantities (I). *Fuzzy Sets System*.

[72] Chiao K.-P. A new ranking approach for general interval type-2 fuzzy sets using extended alpha cuts representation.

[73] Yager R. R. (1980). On a general class of fuzzy connectives. *Fuzzy Sets and Systems*.

[74] Chen S.-J., Chen S.-M. (2007). Fuzzy risk analysis based on the ranking of generalized trapezoidal fuzzy numbers. *Applied Intelligence*.

[75] Liang C., Wu J., Zhang J. (2006). *Ranking Indices and Rules for Fuzzy Numbers Based on Gravity Center Point*.

[76] Wang Y.-J., Lee H.-S. (2008). The revised method of ranking fuzzy numbers with an area between the centroid and original points. *Computers & Mathematics with Applications*.

[77] Shieh B. S. (2007). An approach to centroids of fuzzy numbers. *International Journal of Fuzzy Systems*.

[78] Wang Y.-M., Yang J.-B., Xu D.-L., Chin K.-S. (2006). On the centroids of fuzzy numbers. *Fuzzy Sets and Systems*.

[79] Figueroa-Garcia J. C., Chalco-Cano Y., Roman-Flores H. (2018). Yager index and ranking for interval type-2 fuzzy numbers. *IEEE Transactions on Fuzzy Systems*.

[80] Opricovic S., Tzeng G.-H. (2004). Compromise solution by MCDM methods: a comparative analysis of VIKOR and TOPSIS. *European Journal of Operational Research*.

[81] Chen L. Y., Wang T.-C. (2009). Optimizing partners’ choice in IS/IT outsourcing projects: the strategic decision of fuzzy VIKOR. *International Journal of Production Economics*.

[82] Opricovic S., Tzeng G.-H. (2007). Extended VIKOR method in comparison with outranking methods. *European Journal of Operational Research*.

[83] Wei J., Lin X. The multiple attribute decision-making VIKOR method and its application.

[84] [Internet] BLOOMBERG China seeks plasma from recovered patients as virus treatment. https://time.com/5784286/covid-19-chinaplasma-%20treatment/.

[85] Kreil T. R., Farcet M. R. (2018). Immunoglobulins and virus antibody titers: of past needs, current requirements, and future options. *Transfusion*.

[86] Shen C., Wang Z., Zhao F. (2020). Treatment of 5 critically ill patients with COVID-19 with convalescent plasma. *JAMA*.

[87] Bryner J. Flu drug used in Japan shows promise in treating COVID-19. http://www.Livesicience.com.

